The article "Tert-butylhydroquinone lowers blood pressure in AngII-induced hypertension in mice via proteasome-PTEN-Akt-eNOS pathway" was retracted in 2019. Reasons: duplicated images; concerns about the data.

# Tert-butylhydroquinone lowers blood pressure in AngII-induced hypertension in mice via proteasome-PTEN-Akt-eNOS pathway

**DOI:** 10.1038/srep29589

**Published:** 2016-07-20

**Authors:** Bing-Can Xu, Hui-Bao Long, Ke-Qin Luo

**Affiliations:** 1 Department of Emergency, Sun Yat-Sen Memorial Hospital, Sun Yat-Sen University, Guangzhou, China

## Abstract

Tert-butylhydroquinone (tBHQ), as an antioxidant, has been widely used for many years to prevent oxidization of food products. The aim of this study was to investigate whether tBHQ activates endothelial nitric oxide synthase (eNOS) to prevent endothelial dysfunction and lower blood pressure. The role of Akt in tBHQ-induced eNOS phosphorylation was examined in human umbilical vein endothelial cells (HUVEC) or in mice. tBHQ treatment of HUVEC increased both Akt-Ser473 phosphorylation, accompanied with increased eNOS-Ser1177 phosphorylation and NO release. Mechanically, pharmacologic or genetic inhibition of Akt abolished tBHQ-enhanced NO release and eNOS phosphorylation in HUVEC. Gain-function of PTEN or inhibition of 26S proteasome abolished tBHQ-enhanced Akt phosphorylation in HUVEC. *Ex vivo* analysis indicated that tBHQ improved Ach-induced endothelium-dependent relaxation in LPC-treated mice aortic arteries, which were abolished by inhibition of Akt or eNOS. In animal study, administration of tBHQ significantly increased eNOS-Ser1177 phosphorylation and acetylcholine-induced vasorelaxation, and lowered AngII-induced hypertension in wildtype mice, but not in mice deficient of Akt or eNOS. In conclusion, tBHQ via proteasome-dependent degradation of PTEN increases Akt phosphorylation, resulting in upregulation of eNOS-derived NO production and consequent improvement of endothelial function *in vivo*. In this way, tBHQ lowers blood pressure in hypertensive mice.

Loss of nitric oxide (NO) produced by endothelial nitric oxide synthase (eNOS) is essential for endothelial dysfunction, defined by impaired endothelium-dependent relaxation, which is an early marker for cardiovascular diseases (CVD), such as hypertension^1^. Many of the risk factors of CVD including hyperglycemia, dyslipidemia, hyperhomocysteinemia, and angiotensin II (AngII) can decrease NO production and induce the pathogenesis of hypertension^2^,^3^. Previous studies showed that the phosphorylation of eNOS at serine 1177 plays an important role in the generation of NO in endothelial cells^4^,^5^. Activations of eNOS upstream kinase, such as Akt and AMP-activated protein kinase, increase phosphorylation of eNOS and improve endothelial function^6^. However, better understanding of regulation of eNOS upstream kinase responsible for endothelial dysfunction remains largely unknown, limiting effective therapeutic interventions on CVD.

The article "Tert-butylhydroquinone lowers blood pressure in AngII-induced hypertension in mice via proteasome-PTEN-Akt-eNOS pathway" was retracted in 2019. Reasons: duplicated images; concerns about the data.

Tert-butylhydroquinone (tBHQ) is a synthetic phenolic antioxidant, widely used as a food preservative to extend the shelf life of food^7^. A rich body of evidence has demonstrated that tBHQ is effective in protecting against cellular dysfunction induced by oxidative stress inducers, such as alcohol, dopamine, hydrogen peroxide, and glutamate, in various cell types^7^. Recently, it was reported that *t*-BHQ activated Akt, which ameliorates pressure overload-induced cardiac dysfunction^8^ or produce antioxidant response in rat hepatoma cell line^9^.

Available data suggest that deficiency of NO mediated endothelial dysfunction in AngII-induced hypertensive mice, as well as in experimental hypercholesterolemia pig^10^. It remained to be reasonably established if treatment of tBHQ via Akt increase eNOS-derived NO production in AngII-induced endothelial dysfunction. Here we report that tBHQ activates Akt resulting in phosphorylation of eNOS and consequent reduction of AngII-induced hypertension in mice.

## Methods and Materials

### Materials

tBHQ, MG132 (Z-Leu-Leu-Leu-CHO), lysophosphatidylcholine (LPC), wortmannin, NG-Nitro-L-arginine Methyl Ester (L-NAME), acetylcholine (Ach), phenylephrine (PE), sodium nitroprusside (SNP), angiotensin II (AngII) were obtained from Sigma (St. Louis, MO). 4-Amino,5-aminomethyl-2′,7′-difluorescein (DAF) was obtained from Cayman Chemical Company (Ann Arbor, Michigan, USA). Antibodies against PTEN (Cat, #9188), Akt (Cat, #4691), phospho-Akt-Ser^473^ (Cat, #5012), eNOS (Cat, #9586), phospho-eNOS-Ser^1177^ (Cat, #9575), phospho-eNOS-Ser^113^ (Cat, #9575), phospho-eNOS-Thr^495^ (Cat, #9574,), and β-actin (Cat, #3700) were obtained from Cell Signaling Technology (Beverly, MA). Control and Akt siRNAs were from Santa Cruz Biotechnology Inc. (Santa Cruz, CA). The siRNA delivery agent, Lipofectamine 2000, was from Invitrogen (Carlsbad, CA).

### Animals

Wild-type (*WT*, C57B16) mice and gene knockout of Akt (*Akt*^−/−^) or eNOS (*eNOS*^−/−^) mice, 8–12 weeks of age, 20–25 g, were obtained from the Jackson Laboratory (Bar Harbor, ME). Mice were housed in temperature-controlled cages with a 12-h light-dark cycle and given free access to water chows. Mice were fed with normal diet containing tBHQ a ratio of 1% (w/w) for 2 weeks days prior to AngII infusion for another 14 days. This animal study was carried out in strict accordance with the recommendations in the Guide for the Care and Use of Laboratory Animals of the National Institutes of Health. The animal protocol was reviewed and approved by Sun Yat-Sen University, Institute of Animal Care and Use Committee.

The article "Tert-butylhydroquinone lowers blood pressure in AngII-induced hypertension in mice via proteasome-PTEN-Akt-eNOS pathway" was retracted in 2019. Reasons: duplicated images; concerns about the data.

### Cell culture

Human umbilical vein endothelial cells (HUVEC) were obtained from Clonetics Inc. (Walkersville, MD) and cultured as describe previously^11^. HUVECs were grown in endothelial basal medium supplemented with 2% fetal bovine serum and penicillin (100 u/ml), and streptomycin (100 μg/ml). Cultured cells were used between passages 3 and 8. All cells were incubated in a humidified atmosphere of 5% CO_2_ + 95% air at 37 °C. When 70–80% confluent, the cells were treated with different agents.

### Adenovirus infection to HUVEC

HUVECs were infected with ad-vector or ad-PTEN-CA in medium with 2% FCS overnight. The cells were then washed and incubated in fresh endothelium growth medium without FCS for an additional 12 h before experimentation.

### Transfection of siRNA into cells

Transient transfection of siRNA was carried out according to Santa Cruz’s protocol^12^. Briefly, the siRNAs were dissolved in siRNA buffer (20 mM KCl; 6 mM HEPES, pH 7.5; 0.2 mM MgCl_2_) to prepare a 10 μM stock solution. Cells grown in 6-well plates were transfected with siRNA in transfection medium containing liposomal transfection reagent (Lipofectamine RNAiMax, Invitrogen, Shanghai branch, China). For each transfection, 100 μl transfection medium containing 4 μl siRNA stock solution was gently mixed with 100 μl transfection medium containing 4 μl transfection reagent. After 30-min incubation at room temperature, siRNA-lipid complexes were added to the cells in 1.0 ml transfection medium, and cells were incubated with this mixture for 6 h at 37 °C. The transfection medium was then replaced with normal medium, and cells were cultured for 48 h.

### Western blot analysis

Cells and thawed mouse aortas were lysed in cold RIPA buffer. Protein concentrations were determined with a bicinchoninic acid protein assay system (Pierce, Rockford, IL). Proteins were subjected to Western blots using ECL-Plus, as described previously^13^. The intensity (area X density) of the individual bands on Western blots was measured by densitometry (model GS-700, Imaging Densitometer; Bio-Rad). The background was subtracted from the calculated area and the control group was set as 100%.

### eNOS activity assay

eNOS activity was monitored by L-[^3^H]citrulline production from L-[^3^H]arginine as described previously^11^. Briefly, protein samples were incubated in reaction buffer containing 1 mM L-arginine, 100 mM NADPH, 1 mM tetrahydrobiopterin, 0.2 μCi of L-[^3^H]arginine (>66 Ci/mmol), and Nω-hydroxy-nor-L-arginine (10 μM). The reaction was performed at 37 °C for 15 min and the mixture was separated by Dowex-50W ion-exchange chromatography in 20 mM HEPES (pH 5.5), 2 mM EDTA, and 2 mM EGTA, and the flow-through was used for liquid scintillation counting.

The article "Tert-butylhydroquinone lowers blood pressure in AngII-induced hypertension in mice via proteasome-PTEN-Akt-eNOS pathway" was retracted in 2019. Reasons: duplicated images; concerns about the data.

### Measurement of NO production

For NO detection, cells grown in 24-well plates were incubated for 30 min in the presence of 10 μM DAF in PBS in the dark at 37 °C. Cells were then washed with PBS to remove excessive DAF, and the change in fluorescence was recorded for 15 min at room temperature using a microplate reader (FL 600, Bio-Tek) with the excitation wavelength set at 485 nm and the emission wavelength set at 530 nm. Changes in fluorescence were also visualized with a fluorescence microscope (Olympus IX71), and images were captured for analysis^14^. The intensity of DAF fluorescence was read by microplate reader.

NO level in serum or in isolated mice aorta was assayed by the Griess method as described previously^15^. Because NO is a compound with a short half-life and is rapidly converted to the stable end products nitrate (NO_3_^−^) and nitrite (NO_2_^−^), the principle of the assay is the conversion of nitrate into nitrite by cadmium and followed by color development with Griess reagent (sulfanilamide and *N*-naphthyl ethylenediamine) in acidic medium. The total nitrite was measured by Griess reaction. The absorbance was determined at 540 nm with a spectrophotometer.

### 26S proteasome activity assay

Cells were washed with PBS and then with buffer I (50 mM Tris, pH 7.4, 2 mM DTT, 5 mM MgCl_2_, 2 mM ATP). The cells were then made into pellets by centrifugation. Homogenization buffer (50 mM Tris, pH 7.4, 1 mM DTT, 5 mM MgCl_2_, 2 mM ATP, 250 mM sucrose) was added, and cells were subjected to a vortex for 1 minute. Cell debris was removed by centrifugation at 1000 g for 5 minutes followed by 10000 g for 20 minutes. Protein (100 μg) from each sample was diluted with buffer I to a final volume of 1000 μl. The fluorogenic proteasome substrate Suc-LLVY-7-amido-4-methylcoumarin was added at a final concentration of 80 μM in 1% DMSO. Cleavage activity was monitored continuously by detection of free 7-amido-4-methylcoumarin with a fluorescence plate reader (Gemini, Molecular Devices, Sunnyvale, CA, USA) at 380/460.

### Reverse-transcription polymerase chain reaction for PTEN

RNA was isolated from the treated HUVECs with the total RNA isolation protocol for the RNeasy Mini Kit (Qiagen Inc, Valencia, Calif). Reverse-transcription polymerase chain reaction was performed according to the manufacturer’s protocol. The procedures for semiquantitative reverse transcription–polymerase chain reaction (RT-PCR) were as described using forward (5′-GCCATGCAGTTCTTCACCAA-3′) and reverse (5′-AGGCTTCCGTGATTGCTACA-3′) primers corresponding to human PTEN mRNA. Reactions were run for 30 cycles at conditions as follows: denaturation for 30 seconds at 94 °C, annealing for 30 seconds at 57 °C, and extension for 30 seconds at 72 °C. Constitutively expressed GADPH mRNA was amplified with forward (5′-ACCACAGTCCATGCCATCACTGCC-3′) and reverse (5′-ACCAGGAAATGAG CTTGACAAAGT-3′) primers in a similar manner for 26 cycles.

The article "Tert-butylhydroquinone lowers blood pressure in AngII-induced hypertension in mice via proteasome-PTEN-Akt-eNOS pathway" was retracted in 2019. Reasons: duplicated images; concerns about the data.

### Measurement of tension development in aortic rings

Organ chamber study was performed as described previously^11^,^16^,^17^,^18^. Mice were sacrificed under anesthesia by intravenous injection with pentobarbital sodium (30 mg/kg). The descending aorta isolated by removing the adhering perivascular tissue carefully was cut into rings (3–4 mm in length). Aortic rings were suspended and mounted to organ chamber by using two stainless. The rings were placed in organ baths filled with Kreb’s buffer of the following compositions (in mM): NaCl, 118.3; KCl, 4.7; MgSO_4_, 0.6; KH_2_PO_4_, 1.2; CaCl_2_, 2.5; NaHCO_3_, 25.0; EDTA, 0.026; pH 7.4 at 37 °C and gassed with 95% O_2_ plus 5% CO_2_, under a tension of 0.8 g, for 90-minute equilibration period. During this period, the Kreb’s solution was changed every 15 min. After the equilibration, aortic rings were challenged with 60 mM KCl. After washing and another 30 minutes equilibration period, contractile response was elicited by PE (1 μM). At the plateau of contraction, accumulative Ach or SNP was added into the organ bath to induce vessel relaxation.

### Blood pressure measurement

Blood pressure was determined by radiotelemetry methods as described previously^19^,^20^. Under anaesthesia (pentobarbital sodium, 30 mg/kg, I.P.), mice were implanted with a TA11PA-C10 radiotelemetry transmitter (Data Sciences, Laurel, Md) for 24-hour recording of arterial pressure and heart rate with a radiotelemetry data-acquisition program (Dataquest ART 3.1, Data Sciences). Hemodynamic measurements were sampled for 10 seconds every 10 minutes. Data were reported as 24-hour average.

### Statistical analysis

Statistical comparisons of vasodilation were performed using a two-way ANOVA. Intergroup differences were analyzed using Bonferroni’s post test. Analysis of time-course studies was performed with repeated measures ANOVA. All other results were analyzed with one-way ANOVA. Values are expressed as mean ± SEM. *P* values less than 0.05 were considered as significant.

## Results

### tBHQ increases Akt phosphorylation in cultured endothelial cells

tBHQ has been reported to activate Akt in many cells, such as liver cell, cancer cell, and neuron cell^7^. To investigate whether tBHQ also activates Akt in endothelial cells, confluent HUVEC were treated with varying concentrations of tBHQ for 0.5 to 24 h. Akt activation was indirectly assessed by western blot analysis of Akt phosphorylation at Ser473, which is essential for Akt activity^21^. As shown in Fig. 1A, the phosphorylation of Akt gradually increased beginning from 1 h after incubation with 50 μM of tBHQ and reached peak levels at 12 hs in cells. tBHQ treatment did not alter total levels of Akt, suggesting that tBHQ-induced phosphorylation of Akt was not due to altered expression of the total protein.

The article "Tert-butylhydroquinone lowers blood pressure in AngII-induced hypertension in mice via proteasome-PTEN-Akt-eNOS pathway" was retracted in 2019. Reasons: duplicated images; concerns about the data.

We next examined the dose-dependent effects of tBHQ on Akt-Ser473 phosphorylation. tBHQ did not affect phosphorylation of Akt at a concentration of 5 μM (Fig. 1B). In contrast, tBHQ at 25 μM significantly enhanced Akt phosphorylation. Increasing concentrations of tBHQ (50 and 100 μM) further enhanced Akt phosphorylation. Levels of total Akt remained unchanged at all tBHQ concentrations tested. Based on these results, 50 μM was selected to stimulate HUVEC for 12 hs in subsequent experiments.

### tBHQ increases eNOS phosphorylation and activity in endothelial cells

The important function of endothelial cell is to generate eNOS-derived NO to regulate vascular tone^15^. To investigate whether tBHQ activates eNOS, we measured the eNOS phosphorylation at Ser1177, which represents active eNOS in endothelial cells^4^. As shown in Fig. 1A,C, treatment of HUVEC with tBHQ increased eNOS-Ser1177 phosphorylation and activity in time-course. The dose-dependent effects of tBHQ on eNOS phosphorylation and activity (Fig. 1B,D) were also similar to those for Akt phosphorylation. tBHQ treatment did not alter total levels of eNOS, indicating that tBHQ-induced phosphorylation of eNOS was not due to altered expression of the total protein.

We also detected the effects of tBHQ in HUVEC under AngII stimulation. As shown in Fig. 1E, tBHQ increased both Akt and eNOS-Ser1177 phosphorylations in HUVEC treated with or without AngII. The effects of tBHQ on increasing eNOS and Akt phosphorylations were much stronger than in basal condition, indicating that tBHQ may protect endothelial cells functions under stress.

Besides serine 1177, other point of phosphorylation may modulate eNOS activity, such as Thr495 and Ser113^22^,^23^. Thus, we detected the effect of tBHQ on these sites. As indicated in Fig. 1F, we did not see any alterations of the sites phosphorylations. This suggests us that eNOS phosphorylation at Ser1177, but not Thr495 and Ser113, plays a major role in the effects of tBHQ.

### tBHQ-induced eNOS phosphorylation is Akt-dependent

Previously studies have demonstrated that Akt directly phosphorylates and activates eNOS in endothelial cells^24^. Given that tBHQ activates both Akt and eNOS in HUVEC, we then investigated whether the tBHQ-stimulated eNOS phosphorylation involves Akt in HUVEC by silence of Akt gene expression with specific siRNA transfection. As shown in Fig. 2A, transfection of Akt siRNA but not control siRNA markedly abolished tBHQ-induced eNOS phosphorylation in HUVEC. Consistent with these results, siRNA-mediated knockdown of Akt abolished tBHQ-enhanced NO production and eNOS activity, while control siRNA had no effects (Fig. 2B–D). Collectively, it suggests that Akt is required tBHQ-stimulated eNOS phosphorylation and NO productions in endothelial cells.

The article "Tert-butylhydroquinone lowers blood pressure in AngII-induced hypertension in mice via proteasome-PTEN-Akt-eNOS pathway" was retracted in 2019. Reasons: duplicated images; concerns about the data.

### PTEN is essential to tBHQ-induced Akt phosphorylation

To begin to understand how tBHQ activates Akt, we investigated whether tBHQ changes PTEN, a lipid phosphatase that dephosphorylates Akt^25^. As shown in Fig. 3A,B, tBHQ reduced total protein levels of PTEN in time- or dose-dependent manner. Importantly, tBHQ-induced Akt phosphorylation was blocked by overexpression of PTEN in cells infected with adenovirus containing PTEN cDNA, but not vector (Fig. 3C). Taken together, these results imply that tBHQ-induced Akt phosphorylation requires PTEN.

### The 26S proteasome mediates the tBHQ-induced reduction of PTEN in cells

The levels of PTEN protein are controlled by 26S proteasome-mediated degradation^26^. Thus, we investigated whether tBHQ via activation of 26S proteasome increases PTEN protein degradation in HUVEC. As expected, tBHQ dramatically increased 26S proteasome in endothelial cells, while MG132, a positive proteasome inhibitor, inhibited 26S proteasome activity (Fig. 4A).

To determine the role of 26S proteasome in tBHQ-reduced PTEN protein stability, we treated cells with MG132 plus tBHQ. As indicated in Fig. 4B, co-administration of MG132 abolished tBHQ-induced reduction of PTEN protein. Both tBHQ and MG132 or plus had no effects on PTEN mRNA levels (Fig. 4C). All these data suggest that the alteration of PTEN level is due to the activation of the 26S proteasome by tBHQ.

### tBHQ preserves endothelium-dependent relaxation impaired by LPC in isolated mice aortic rings

Deficiency of eNOS-derived NO, as a major component to endothelium-dependent relaxation factor, is an early marker for endothelial dysfunction in CVD^1^,^3^,^11^,^12^. We then performed *ex vivo* experiments to test whether activation of Akt-eNOS pathway by tBHQ prevents endothelial dysfunctions by incubating isolated mice aortic rings with LPC, which is the major metabolite of ox-LDL, a common risk factor for CVD. In basal condition, tBHQ had no effects on Ach-induced endothelium-dependent relaxation (Fig. 5A), indicating that tBHQ did not affect endothelial function, although tBHQ has direct and indirect redox effects. However, exposure of aortic rings to LPC dramatically impaired Ach-induced endothelium-dependent relaxation (Fig. 5B). Further, tBHQ dose-dependently reversed Ach-induced endothelium-dependent relaxation in aortic rings incubated with LPC (Fig. 5B), suggesting that tBHQ functions as a protector on vascular endothelium.

The article "Tert-butylhydroquinone lowers blood pressure in AngII-induced hypertension in mice via proteasome-PTEN-Akt-eNOS pathway" was retracted in 2019. Reasons: duplicated images; concerns about the data.

### Inhibition of Akt or eNOS attenuates LPC-induced impairment of endothelium-dependent relaxation *ex vivo*

The role of Akt or eNOS on tBHQ-prevented endothelial dysfunctions induced by LPC was next determined. As shown in Fig. 5C,D, preincubation of mice aortic rings with either wortmannin (1 μM) of Akt inhibitor or L-NAME (1 mM) of eNOS inhibitor partially bypassed tBHQ-improved Ach-induced endothelium-dependent relaxation and NO productions in LPC-treated mice aortic rings.

Because both wortmannin at 1 μM and L-NAME at 1 mM did not completely reversed the effects of tBHQ, we increased the concentrations of wortmannin to 5 μM and L-NAME to 5 mM. As indicated in Fig. 5E, high concentrations of wortmannin and L-NAME totally blocked the protective effects of tBHQ on LPC-induced endothelial dysfunction. However, both inhibitors further decreased the NO productions (Fig. 5F). Taking these data together, it demonstrates that tBHQ improves endothelial functions, which is possibly related to Akt-eNOS signaling.

### Administration of tBHQ prevents AngII-induced endothelial dysfunction in *WT* mice

We next determine the effects of tBHQ on endothelial dysfunction *in vivo*. The model of endothelial dysfunction model was established by AngII infusion as described previously^2^. As indicated in Fig. 6A, infusion of AngII dramatically decreased Ach-induced endothelium-dependent vasorelaxation in *WT* mice, consistent with other’s reports. Administration of tBHQ rescued AngII-induced impairments of endothelium-dependent relaxation. In addition, SNP-induced endothelium-independent relaxation was not altered in all groups (Fig. 6B), indicating that the effects of tBHQ is limited to vascular endothelium, but not smooth muscle.

### Role of Akt in tBHQ-enhanced endothelium-dependent vasorelaxation in mice

Next, to investigate the role of Akt in endothelial function, we tested the effect of tBHQ in *Akt*^−/−^ mice. As indicated in Fig. 6C, Ach-induced vasodilatation was markedly attenuated in *Akt*^−/−^ mice. It should be noted that, following treatment with tBHQ, Ach-induced vasodilatation in aortic arteries of *Akt*^−/−^ mice was not improved by tBHQ, compared to *WT* mice (Fig. 6A). SNP-induced endothelium-independent relaxation was identical in each group in *Akt*^−/−^ mice (Fig. 6D). Taking these data together, it indicates that Akt plays an important role in enhanced endothelial function elicited by tBHQ.

The article "Tert-butylhydroquinone lowers blood pressure in AngII-induced hypertension in mice via proteasome-PTEN-Akt-eNOS pathway" was retracted in 2019. Reasons: duplicated images; concerns about the data.

### tBHQ lowers AngII-induced systemic hypertension in mice

Endothelial dysfunction contributes to the pathophysiology of hypertension^1^. We then investigated whether tBHQ lowers blood pressure in hypertensive model. Mice were implanted with osmatic pump filling with AngII to establish hypertensive model as described previously^27^. Systemic BP was measured by radio telemetry method. As shown in Fig. 7A,B, both systolic BP and diastolic BP began to increase at 2^nd^ day and reached to the high level at the 6–14^th^ day after AngII infusion. Administration of mice with tBHQ remarkably suppressed AngII-induced increases of systolic BP and diastolic BP, indicating that tBHQ is effective to lower blood pressure *in vivo*.

### Deletion of Akt abolishes the effects of lowering BP induced by tBHQ in AngII-infused mice

To examine the role of Akt in tBHQ-induced reduction of blood pressure in AngII-infused mice, we also determined the effects of tBHQ in in *Akt*^−/−^ mice. In contrast to WT mice, the increased systolic BP and diastolic BP were not normalized by tBHQ (Fig. 7C,D) while Akt is deficient in mice. These data demonstrate that Akt activation is involved in tBHQ-induced effects on lowering BP *in vivo*.

### tBHQ via eNOS lowers BP in acute hypertensive mice induced by AngII

It has been known and eNOS depletion results in spontaneous hypertension^28^,^29^,^30^,^31^. Thus, we analyzed the role of eNOS on systemic blood pressures lowered by tBHQ. As shown in Fig. 7E,F, both sBP and dBP were significantly elevated in eNOS-null mice, compared to those in *WT* animals (Fig. 7A,B). As expected, administration of tBHQ did not alter sBP and dBP in eNOS-null mice, indicating that eNOS is required for in tBHQ-reduced systemic BPs in mice.

### tBHQ increases eNOS phosphorylation and NO production *in vivo*, which is Akt dependent

Finally, we determined the effects of tBHQ on p-Akt, p-eNOS and NO production *in vivo*. As shown in Fig. 8A,B, aortic levels of eNOS phosphorylation, Akt phosphorylation and serum levels of NO were significantly elevated in tBHQ-treated *WT* but not *Akt*^−/−^ mice infused with AngII. Overall, these results suggest that Akt is required for tBHQ-enhanced eNOS-NO pathway *in vivo*.

## Discussion

In the present study, we have for the first time provided evidences that tBHQ via PTEN-dependent Akt activation increases NO release and improves endothelial function *in vivo*. Furthermore, we have characterized that activation of proteasome mediates the protective effects of tBHQ in endothelial cells. These findings support a key role of proteasome-PTEN-Akt-eNOS-NO pathway in the anti-hypertensive effects of tBHQ *in vivo*.

tBHQ is a synthetic phenolic antioxidant, widely used as a food preservative to extend the shelf life of food. A rich body of evidence has demonstrated that tBHQ is effective in protecting against cellular dysfunction induced by oxidative stress inducers, such as alcohol, dopamine, hydrogen peroxide, and glutamate, in various cell types^32^,^33^,^34^. tBHQ has been extensively studied and is known to exhibit multiple pharmacological activities such as antidiabetic, anti-inflammatory, neuroprotective, and antiproliferative activities in combating against diabetes and cancer^35^,^36^,^37^,^38^. The present study further indicates the effects of anti-hypertension of tBHQ. Our results may extent the clinical application of tBHQ in the management of hypertension which related to hyperlipidemia, insulin resistance, metabolic syndrome, and type 2 diabetes from preclinical and clinical trials.

The article "Tert-butylhydroquinone lowers blood pressure in AngII-induced hypertension in mice via proteasome-PTEN-Akt-eNOS pathway" was retracted in 2019. Reasons: duplicated images; concerns about the data.

Mechanically, the anti-hypertensive effects if tBHQ is mediated by Akt-dependent eNOS activation. It has been well-established that tBHQ exerts its protective effects through a mechanism whereby it increases nuclear factor like 2 protein stability via inhibition of the Keap1-mediated ubiquitination^9^,^39^,^40^. In this study, we observed that tBHQ increased proteasome activity to induce PTEN degradation. This raised subsequent reduction of Akt dephosphorylation and eNOS activation in endothelial cells and VSMCs. In this way, tBHQ produces the effects of anti-hypertension via NO release from endothelium. Our results strongly imply that an activation of Akt by tBHQ in endothelial cells dependent on PTEN, in consistent with previous reports^35^, which tBHQ via PI3K activates Akt. This discrepancy should be explained by the different cell types. In endothelial cell, PYEN might play a dominant role in the regulation of Akt phosphorylation by tBHQ. Indeed, Ping *et al* has reported that PTEN-mediated Akt dephosphorylation is a key contributing to endothelial insulin resistance^41^,^42^,^43^.

We also show that the reduction of PTEN by tBHQ is due to the degradation by proteasome. The ubiquitin proteasome system acts to fine tune the intracellular levels of these factors to maintain optimal cell division, growth, differentiation, signal transduction, and stress responses. It plays a key role in protein quality by removing damaged, oxidized, and/or misfolded proteins. Structurally, the proteasome is comprised of a catalytic core, the 20S proteasome, and a multisubunit regulatory protein, termed PA700, which confers ATP/ubiquitin-dependent proteolytic properties to the proteasome^44^. The proteasome can also degrade proteins in an ATP-dependent and ubiquitin-independent fashion^45^. Proteasome-dependent degradation of PTEN, in particular, might be essential for the effects of tBHQ in regulation of endothelial function, as it decreases Akt phosphorylation at serine 473, which is a key site for its activity to regulate eNOS phosphorylation^4^,^5^ and NO production. Further studies should focus on the regulation of tBHQ on proteasome activity.

The article "Tert-butylhydroquinone lowers blood pressure in AngII-induced hypertension in mice via proteasome-PTEN-Akt-eNOS pathway" was retracted in 2019. Reasons: duplicated images; concerns about the data.

A limitation of this study is that both wortmannin and L-NAME at low concentration did not completely reverse the effects of tBHQ on LPC-induced endothelial dysfunction. Thus, we increased the concentrations of them and observed that they completely blocked tBHQ’s effects, indicating tBHQ via an Akt-eNOS-dependent pathway improves endothelial function. In facts, some inhibitor may produce off-target effects. As a proteasome inhibitor, the effects of MG132 on endothelial function is so controversial, for example, it has been reported that MG132 induces apoptosis and endoplasmic reticulum stress^19^,^46^. However, Wang S *et al*. reported that MG132 inhibits degradation of IκBα or GTPCH to suppress oxidative stress in endothelial cells^3^,^12^. Besides, the concentration of tBHQ given in a ratio of 1% (w/w) to hypertensive mice is a little high. Although the upper limit set by the FDA is 0.02% of the oil or fat content in foods, the dose is set for human. According to Chodera’s report^47^, the pharmacodynamic properties are different in human and mice. This is why a ratio of 1% (w/w) to hypertensive mice was chosen by us.

In summary, we have uncovered a novel pathway by which the tBHQ prevents endothelial dysfunction and lowers blood pressure in hypertensive mice. This pathway, which relies on PTEN as a mediator of Akt activation, stimulates NO production through eNOS phosphorylation. Although the possible carcinogenic effects might be produced by tBHQ^48^, our results indicate that PTEN-Akt pathway may help account for the beneficial effects of tBHQ on endothelial function and hypertension.

## Additional Information

**How to cite this article**: Xu, B.-C. *et al*. Tert-butylhydroquinone lowers blood pressure in AngII-induced hypertension in mice via proteasome-PTEN-Akt-eNOS pathway. *Sci. Rep.* **6**, 29589; doi: 10.1038/srep29589 (2016).

## Figures and Tables

**Figure 1:** tBHQ activates eNOS and Akt in HUVEC. (**A**) HUVEC were treated with 50 μM tBHQ for the indicated times. The levels of Akt and eNOS phosphorylations in total cell lysates were analyzed by western blot. The blot is a representative of three blots obtained from separated experiments. Data presented are means ± SEM from 3 independent experiments. *P < 0.05 vs. control group (point 0). (**B**) HUVEC were treated with varying concentrations of tBHQ for 12 hours. The levels of Akt and eNOS phosphorylations in total cell lysates were analyzed by western blot. The blot is a representative of three blots obtained from separated experiments. Data presented are means ± SEM from 3 independent experiments. *P < 0.05 vs. control group (point 0). (**C**) eNOS activity was assessed by citrulline assay in (**A)**. (**D**) eNOS activity was assessed by citrulline assay in (**B)**. (**E**) HUVEC were pretreated with tBHQ (50 μM) for 30 minutes followed by AngII (1 μM) for 12 hours. Total cell lysates were analyzed by western blot for the indicated proteins. Data presented are means ± SEM from 3 independent experiments. *P < 0.05 vs. vehicle alone. ^#^*P* < 0.05 vs. tBHQ alone. (**F**) HUVEC were treated with tBHQ (50 μM) for 12 hours. Total cell lysates were analyzed by western blot for the indicated proteins. The blot is a representative of three blots obtained from separated experiments.

The article "Tert-butylhydroquinone lowers blood pressure in AngII-induced hypertension in mice via proteasome-PTEN-Akt-eNOS pathway" was retracted in 2019. Reasons: duplicated images; concerns about the data.

**Figure 2:** Akt mediates tBHQ-induced eNOS phosphorylation and NO production in cultured endothelial cells. (**A**) HUVEC were infected with control or Akt siRNA for 48 hours. Then cells were exposed to tBHQ at 25 μM for 6 hours. Total cell lysates were analyzed by western blot for the indicated proteins. The blot is a representative of four blots obtained from four separated experiments. Data presented are means ± SEM from 4 independent experiments. *P < 0.05 vs. control group. ^#^*P* < 0.05 vs. control siRNA alone. NS indicates no significance. (**B–D**) HUVEC infected with control or Akt siRNA for 48 hours. The NO production was determined by measuring the intensity of DAF fluorescence in (**B)** and quantitative analysis of NO amount was shown in (**C)**. Total cell lysates were subject to assay eNOS activity (**D**). Data presented are means ± SEM from 4 independent experiments. *P < 0.05 vs. control siRNA group. NS indicates no significance.

**Figure 3:** tBHQ induces Akt phosphorylation through PTEN reduction. (**A**) HUVEC were incubated with 25 μM tBHQ for various amounts of time. After the appropriate incubation time, cells were lysed and PTEN protein level was measured by western blot. The blot is a representative of four blots obtained from four separated experiments. Data presented are means ± SE from 4 independent experiments. *P < 0.05 vs. control groups. (**B**) HUVEC were treated with varying concentrations of tBHQ for 6 hours. Total cell lysates were analyzed by western blot for the indicated proteins. The blot is a representative of three blots obtained from separated experiments. Data presented are means ± SEM from 3 independent experiments. *P < 0.05 vs. control groups. (**C**) HUVEC were infected with Ad-PTEN-CA or Ad-vector (control) prior to tBHQ stimulation. The blot is a representative of four blots obtained from four separate experiments. Results are expressed as mean ± SEM from four independent experiments. *P < 0.05 vs. control groups. NS indicates no significance.

The article "Tert-butylhydroquinone lowers blood pressure in AngII-induced hypertension in mice via proteasome-PTEN-Akt-eNOS pathway" was retracted in 2019. Reasons: duplicated images; concerns about the data.

**Figure 4:** tBHQ increases 26S-proteasome-dependent PTEN degradation in HUVEC. (**A**) HUVEC were treated with tBHQ (25 μM) or MG132 (1 μM) for 6 hours. 26S proteasome activity was assayed in cell lysates. Results are expressed as mean ± SEM from four independent experiments. *P < 0.05 vs. control groups. (**B**,**C**) HUVEC were treated with tBHQ (25 μM) with or without MG132 (1 μM) for 6 hours. (**B**) The protein level of PTEN was assayed by western blot. (**C**) The mRNA level of PTEN was determined by RT-PCR. Results are expressed as mean ± SEM from four independent experiments. *P < 0.05 vs. control groups. ^#^*P* < 0.05 vs. tBHQ alone. NS indicates no significance.

**Figure 5:** Inhibition of Akt or eNOS by pharmacological reagents abolishes tBHQ-prevented endothelial dysfunction *ex vivo.* (**A**) The isolated mouse aortic rings were incubated with tBHQ (50 μM) for 12 hours and Ach-induced endothelium-dependent relaxation was assayed by organ chamber. (**B**) The isolated mouse aortic rings were preincubated with tBHQ (25, 50, 100 μM) for 30 minutes and then exposed to LPC (4 mg/l) for 2 hours. Ach-induced endothelium-dependent relaxation was assayed by organ chamber. *P < 0.05 vs. control, ^#^*P* < 0.05 vs. LPC. (**C**) Isolated mouse aortic rings were preincubated with tBHQ (50 μM) for 30 minutes with or without wortmannin (1 μM) and L-NAME (1 mM) followed by LPC (4 mg/l) for 2 hours. The endothelium-dependent relaxation induced by acetylcholine was assayed by organ chamber. *P < 0.05 vs. LPC, ^#^*P* < 0.05 vs. tBHQ. (**D**) Isolated mouse aortic rings were preincubated with tBHQ (50 μM) for 30 minutes with or without wortmannin (5 μM) and L-NAME (5 mM) followed by LPC (4 mg/l) for 2 hours. The endothelium-dependent relaxation induced by acetylcholine was assayed by organ chamber. *P < 0.05 vs. LPC, ^#^*P* < 0.05 vs. tBHQ. (**E**) Homogenates of aortic tissues were subjected to measure NO productions by the Griess method in each group. *P < 0.05 vs. Control group. ^#^*P* < 0.05 vs. LPC. ^$^*P* < 0.05 vs. LPC + tBHQ.

**Figure 6:** Deficiency of Akt abrogates tBHQ-induced improvement of endothelial dysfunction in AngII-infused mice. *WT* and *Akt*^−/−^ mice at the age of 8–12 weeks old were fed with normal diet containing tBHQ a ratio of 1% (w/w) for 2 weeks days prior to AngII infusion for another 14 days. Aortas from mice were cut into rings and were mounted in organ chamber to detect vessel bioactivity. The relaxation was induced acetylcholine (Ach) or SNP. (**A**) Endothelium-dependent relaxation of the aortic rings in response to Ach from *WT* mice. (**B**) Endothelium-independent relaxation of the aortic rings in response to SNP from *WT* mice. (**C**) Ach-induced endothelium-dependent relaxation in *Akt*^−/−^ mice. (**D**) SNP-induced endothelium-independent relaxation in *Akt*^−/−^ mice. Each data point represents relaxation expressed as a percentage of the value obtained for phenylephrine-preconstricted aorta. All data were expressed as mean ± SEM. One aortic ring was isolated from each mouse. 10–15 mice in each group. *P < 0.05 vs. Control *WT* or *Akt*^−/−^ group. ^#^*P* < 0.05 vs. AngII in *WT* mice.

The article "Tert-butylhydroquinone lowers blood pressure in AngII-induced hypertension in mice via proteasome-PTEN-Akt-eNOS pathway" was retracted in 2019. Reasons: duplicated images; concerns about the data.

**Figure 7:** tBHQ lowers AngII-induced hypertension in wildtype (*WT*) mice, but not in hypertensive *Akt*^−/−^ mice. *WT, Akt*^−/−^, and *eNOS*^−/−^ mice at the age of 8–12 weeks old were fed with normal diet containing tBHQ a ratio of 1% (w/w) for 2 weeks days prior to AngII infusion. Blood pressure (BP) was monitored by telemetry, as described in Materials and Methods. (**A**) Systolic BP and (**B**) diastolic BP in *WT* mice, (**C**) systolic BP and (**D**) diastolic BP in *Akt*^−/−^ mice, and (**E**) systolic BP and (**F**) diastolic BP in *eNOS*^−/−^ mice were analyzed. Quantitative results are expressed as mean ± SEM. N is 10–15 in each group. *P < 0.05 vs. Control *WT* or *Akt*^−/−^ mice. ^#^*P* < 0.05 vs. AngII mice.

**Figure 8:** tBHQ via Akt activation increases NO production in hypertensive mice. (**A**,**B**) *WT* and *Akt*^−/−^ mice at the age of 8–12 weeks old were fed with normal diet containing tBHQ a ratio of 1% (w/w) for 4 weeks days prior to AngII infusion for 14 days. (**A**) Homogenates of aortic tissues were subjected to perform western blot to assay the levels of P-eNOS and P-Akt. (**B**) Serum NO level was also analyzed by the Griess method. All data were expressed as mean ± SEM. 10–15 mice in each group. *P < 0.05 vs. Control *WT* mice. ^#^*P* < 0.05 vs. AngII mice. NS indicates no significant. (**C**) Proposed mechanism of tBHQ on vascular function.

## References

[b1] WangS. . Acute inhibition of guanosine triphosphate cyclohydrolase 1 uncouples endothelial nitric oxide synthase and elevates blood pressure. Hypertension 52, 484–490 (2008).1864504910.1161/HYPERTENSIONAHA.108.112094PMC3523107

[b2] XuJ., WangS., WuY., SongP. & ZouM. H. Tyrosine nitration of PA700 activates the 26S proteasome to induce endothelial dysfunction in mice with angiotensin II-induced hypertension. Hypertension 54, 625–632 (2009).1959703910.1161/HYPERTENSIONAHA.109.133736PMC2910588

The article "Tert-butylhydroquinone lowers blood pressure in AngII-induced hypertension in mice via proteasome-PTEN-Akt-eNOS pathway" was retracted in 2019. Reasons: duplicated images; concerns about the data.

[b3] WangS., XuJ., SongP., ViolletB. & ZouM. H. *In vivo* activation of AMP-activated protein kinase attenuates diabetes-enhanced degradation of GTP cyclohydrolase I. Diabetes 58, 1893–1901 (2009).1952837510.2337/db09-0267PMC2712774

[b4] DimmelerS. . Activation of nitric oxide synthase in endothelial cells by Akt-dependent phosphorylation. Nature 399, 601–605 (1999).1037660310.1038/21224

[b5] FultonD. . Regulation of endothelium-derived nitric oxide production by the protein kinase Akt. Nature 399, 597–601 (1999).1037660210.1038/21218PMC3637917

[b6] HuL. . Hypoxic preconditioning protects cardiomyocytes against hypoxia/reoxygenation injury through AMPK/eNOS/PGC-1alpha signaling pathway. Int J Clin Exp Pathol 7, 7378–7388 (2014).25550773PMC4270574

[b7] GharaviN., HaggartyS. & El-KadiA. O. Chemoprotective and carcinogenic effects of tert-butylhydroquinone and its metabolites. Current drug metabolism 8, 1–7 (2007).1726651910.2174/138920007779315035

[b8] BaetaB. A. . Characterization of two strains of Anaplasma marginale isolated from cattle in Rio de Janeiro, Brazil, after propagation in tick cell culture. Ticks and tick-borne diseases 6, 141–145 (2015).2546876410.1016/j.ttbdis.2014.11.003

[b9] LiS. . tert-Butylhydroquinone (tBHQ) protects hepatocytes against lipotoxicity via inducing autophagy independently of Nrf2 activation. Biochim Biophys Acta 1841, 22–33 (2014).2405588810.1016/j.bbalip.2013.09.004PMC3884638

[b10] ChadeA. R. . Effects of proteasome inhibition on the kidney in experimental hypercholesterolemia. J Am Soc Nephrol 16, 1005–1012 (2005).1571633110.1681/ASN.2004080674

[b11] WangS., PengQ., ZhangJ. & LiuL. Na+/H+ exchanger is required for hyperglycaemia-induced endothelial dysfunction via calcium-dependent calpain. Cardiovasc Res 80, 255–262 (2008).1859120410.1093/cvr/cvn179

[b12] WangS. . AMPKalpha2 deletion causes aberrant expression and activation of NAD(P)H oxidase and consequent endothelial dysfunction *in vivo*: role of 26S proteasomes. Circ Res 106, 1117–1128 (2010).2016792710.1161/CIRCRESAHA.109.212530PMC2920052

[b13] DavisB. J., XieZ., ViolletB. & ZouM. H. Activation of the AMP-activated kinase by antidiabetes drug metformin stimulates nitric oxide synthesis *in vivo* by promoting the association of heat shock protein 90 and endothelial nitric oxide synthase. Diabetes 55, 496–505 (2006).1644378610.2337/diabetes.55.02.06.db05-1064

[b14] HuH. . Autoinhibitory domain fragment of endothelial NOS enhances pulmonary artery vasorelaxation by the NO-cGMP pathway. Am J Physiol Lung Cell Mol Physiol 286, L1066–1074 (2004).1472951310.1152/ajplung.00378.2003

The article "Tert-butylhydroquinone lowers blood pressure in AngII-induced hypertension in mice via proteasome-PTEN-Akt-eNOS pathway" was retracted in 2019. Reasons: duplicated images; concerns about the data.

[b15] YangX. H. . Rosiglitazone via PPARgamma-dependent suppression of oxidative stress attenuates endothelial dysfunction in rats fed homocysteine thiolactone. J Cell Mol Med 19, 826–835 (2015).2565673510.1111/jcmm.12510PMC4395197

[b16] WangS., LiangB., ViolletB. & ZouM. H. Inhibition of the AMP-activated protein kinase-alpha2 accentuates agonist-induced vascular smooth muscle contraction and high blood pressure in mice. Hypertension 57, 1010–1017 (2011).2146439010.1161/HYPERTENSIONAHA.110.168906PMC3089757

[b17] Shuang-XiW., Li-YingL., HuM. & Yu-HuiL. Na+/H+ exchanger inhibitor prevented endothelial dysfunction induced by high glucose. Journal of cardiovascular pharmacology 45, 586–590 (2005).1590023310.1097/01.fjc.0000161401.14327.38

[b18] WangS. X., XiongX. M., SongT. & LiuL. Y. Protective effects of cariporide on endothelial dysfunction induced by high glucose. Acta pharmacologica Sinica 26, 329–333 (2005).1571592910.1111/j.1745-7254.2005.00042.x

[b19] LiangB. . Aberrant endoplasmic reticulum stress in vascular smooth muscle increases vascular contractility and blood pressure in mice deficient of AMP-activated protein kinase-alpha2 *in vivo*. Arterioscler Thromb Vasc Biol 33, 595–604 (2013).2328816610.1161/ATVBAHA.112.300606PMC3754846

[b20] WangJ., GuoT., PengQ. S., YueS. W. & WangS. X. Berberine via suppression of transient receptor potential vanilloid 4 channel improves vascular stiffness in mice. J Cell Mol Med 19, 2607–2616 (2015).2617734910.1111/jcmm.12645PMC4627566

[b21] MerhiF. . Hyperforin inhibits Akt1 kinase activity and promotes caspase-mediated apoptosis involving Bad and Noxa activation in human myeloid tumor cells. PLoS One 6, e25963 (2011).2199873110.1371/journal.pone.0025963PMC3188562

[b22] GuterbaumT. J. . Endothelial nitric oxide synthase phosphorylation at Threonine 495 and mitochondrial reactive oxygen species formation in response to a high H(2)O(2) concentration. Journal of vascular research 50, 410–420 (2013).2400823610.1159/000354225

[b23] LeeC. H. . CDK5 phosphorylates eNOS at Ser-113 and regulates NO production. J Cell Biochem 110, 112–117 (2010).2021374310.1002/jcb.22515

[b24] RafikovR. . Asymmetric dimethylarginine induces endothelial nitric-oxide synthase mitochondrial redistribution through the nitration-mediated activation of Akt1. J Biol Chem 288, 6212–6226 (2013).2325560810.1074/jbc.M112.423269PMC3585057

[b25] CarneroA. & ParamioJ. M. The PTEN/PI3K/AKT Pathway *in vivo*, Cancer Mouse Models. Front Oncol 4, 252 (2014).2529522510.3389/fonc.2014.00252PMC4172058

[b26] YangL., WangS., SungB., LimG. & MaoJ. Morphine induces ubiquitin-proteasome activity and glutamate transporter degradation. J Biol Chem 283, 21703–21713 (2008).1853959610.1074/jbc.M800809200PMC2490772

The article "Tert-butylhydroquinone lowers blood pressure in AngII-induced hypertension in mice via proteasome-PTEN-Akt-eNOS pathway" was retracted in 2019. Reasons: duplicated images; concerns about the data.

[b27] WangS. . Activation of AMP-activated protein kinase alpha2 by nicotine instigates formation of abdominal aortic aneurysms in mice *in vivo*. Nat Med 18, 902–910 (2012).2256168810.1038/nm.2711PMC3559018

[b28] HuangP. L. . Hypertension in mice lacking the gene for endothelial nitric oxide synthase. Nature 377, 239–242 (1995).754578710.1038/377239a0

[b29] IwakiriY., CadelinaG., SessaW. C. & GroszmannR. J. Mice with targeted deletion of eNOS develop hyperdynamic circulation associated with portal hypertension. Am J Physiol Gastrointest Liver Physiol 283, G1074–1081 (2002).1238152010.1152/ajpgi.00145.2002

[b30] KubisN., RicherC., DomergueV., GiudicelliJ. F. & LevyB. I. Role of microvascular rarefaction in the increased arterial pressure in mice lacking for the endothelial nitric oxide synthase gene (eNOS3pt−/−). J Hypertens 20, 1581–1587 (2002).1217232010.1097/00004872-200208000-00021

[b31] MiyamotoY. . Endothelial nitric oxide synthase gene is positively associated with essential hypertension. Hypertension 32, 3–8 (1998).967463010.1161/01.hyp.32.1.3

[b32] YanD., DongJ., SulikK. K. & ChenS. Y. Induction of the Nrf2-driven antioxidant response by tert-butylhydroquinone prevents ethanol-induced apoptosis in cranial neural crest cells. Biochemical pharmacology 80, 144–149 (2010).2022322510.1016/j.bcp.2010.03.004PMC2860686

[b33] LiJ. . Stabilization of Nrf2 by tBHQ confers protection against oxidative stress-induced cell death in human neural stem cells. Toxicol Sci 83, 313–328 (2005).1552569010.1093/toxsci/kfi027

[b34] LinH. . Activating transcription factor 3 protects against pressure-overload heart failure via the autophagy molecule Beclin-1 pathway. Molecular pharmacology 85, 682–691 (2014).2455013810.1124/mol.113.090092

[b35] KangK. W., ChoM. K., LeeC. H. & KimS. G. Activation of phosphatidylinositol 3-kinase and Akt by tert-butylhydroquinone is responsible for antioxidant response element-mediated rGSTA2 induction in H4IIE cells. Molecular pharmacology 59, 1147–1156 (2001).1130669810.1124/mol.59.5.1147

[b36] BahiaP. K. . Neuroprotective effects of phenolic antioxidant tBHQ associate with inhibition of FoxO3a nuclear translocation and activity. Journal of neurochemistry 123, 182–191 (2012).2280475610.1111/j.1471-4159.2012.07877.xPMC3494983

[b37] SakamotoK., IwasakiK., SugiyamaH. & TsujiY. Role of the tumor suppressor PTEN in antioxidant responsive element-mediated transcription and associated histone modifications. Mol Biol Cell 20, 1606–1617 (2009).1915837510.1091/mbc.E08-07-0762PMC2655256

[b38] XuX. . Wogonin reverses multi-drug resistance of human myelogenous leukemia K562/A02 cells via downregulation of MRP1 expression by inhibiting Nrf2/ARE signaling pathway. Biochemical pharmacology 92, 220–234 (2014).2526427810.1016/j.bcp.2014.09.008

The article "Tert-butylhydroquinone lowers blood pressure in AngII-induced hypertension in mice via proteasome-PTEN-Akt-eNOS pathway" was retracted in 2019. Reasons: duplicated images; concerns about the data.

[b39] LiJ. . Nrf2 protects against maladaptive cardiac responses to hemodynamic stress. Arterioscler Thromb Vasc Biol 29, 1843–1850 (2009).1959246810.1161/ATVBAHA.109.189480PMC12952473

[b40] KasparJ. W., NitureS. K. & JaiswalA. K. Nrf2:INrf2 (Keap1) signaling in oxidative stress. Free radical biology & medicine 47, 1304–1309 (2009).1966610710.1016/j.freeradbiomed.2009.07.035PMC2763938

[b41] SongP. . Thromboxane A2 receptor activates a Rho-associated kinase/LKB1/PTEN pathway to attenuate endothelium insulin signaling. J Biol Chem 284, 17120–17128 (2009).1940352510.1074/jbc.M109.012583PMC2719350

[b42] SongP. . Protein kinase Czeta-dependent LKB1 serine 428 phosphorylation increases LKB1 nucleus export and apoptosis in endothelial cells. J Biol Chem 283, 12446–12455 (2008).1832184910.1074/jbc.M708208200PMC2431011

[b43] SongP. . Reactive nitrogen species induced by hyperglycemia suppresses Akt signaling and triggers apoptosis by upregulating phosphatase PTEN (phosphatase and tensin homologue deleted on chromosome 10) in an LKB1-dependent manner. Circulation 116, 1585–1595 (2007).1787596810.1161/CIRCULATIONAHA.107.716498

[b44] TanakaK. Proteasomes: structure and biology. J Biochem 123, 195–204 (1998).953819210.1093/oxfordjournals.jbchem.a021922

[b45] LamY. A., DeMartinoG. N., PickartC. M. & CohenR. E. Specificity of the ubiquitin isopeptidase in the PA700 regulatory complex of 26 S proteasomes. J Biol Chem 272, 28438–28446 (1997).935330310.1074/jbc.272.45.28438

[b46] TangQ. . Classical swine fever virus NS2 protein promotes interleukin-8 expression and inhibits MG132-induced apoptosis. Virus genes 42, 355–362 (2011).2131823910.1007/s11262-011-0582-z

[b47] ChoderaA. & FellerK. Some aspects of pharmacokinetic and biotransformation differences in humans and mammal animals. Int J Clin Pharmacol Biopharm 16, 357–360 (1978).99374

[b48] GharaviN. & El-KadiA. O. tert-Butylhydroquinone is a novel aryl hydrocarbon receptor ligand. Drug metabolism and disposition: the biological fate of chemicals 33, 365–372 (2005).1560813210.1124/dmd.104.002253

